The article "FoxD2-AS1 promotes glioma progression by regulating miR-185-5P/HMGA2 axis and PI3K/AKT signaling pathway" was retracted in 2023. Reasons: duplicated images; unreliable data; unreliable results or conclusions.

# FoxD2-AS1 promotes glioma progression by regulating miR-185-5P/HMGA2 axis and PI3K/AKT signaling pathway

**DOI:** 10.18632/aging.101843

**Published:** 2019-03-11

**Authors:** Wei Ni, Yaoxiong Xia, Yuxu Bi, Fan Wen, Dong Hu, Lin Luo

**Affiliations:** 1 Department of Neurosurgery, The Third Affiliated Hospital of Kunming Medical University, Kunming 650118, Yunan Province, China; 2 Department of Neurosurgery, Yunnan Cancer Hospital, Kunming 650118, Yunan Province, China; 3 Department of Neurosurgery, Yunnan Cancer Center, Kunming 650118, Yunan Province, China; 4 Department of Radiation Oncology, The Third Affiliated Hospital of Kunming Medical University, Kunming 650118, Yunan Province, China; 5 Department of Radiation Oncology, Yunnan Cancer Hospital, Kunming 650118, Yunan Province, China; 6 Department of Radiation Oncology, Yunnan Cancer Center, Kunming 650118, Yunan Province, China; * Equal contribution

**Keywords:** lncRNA, FOXD2-AS1, glioma, proliferation, metastasis

## Abstract

Background/Aims: The present study was aimed at exploring the role of long noncoding RNA (lncRNA) FOXD2-AS1 in the development and progression of glioma and the underlying mechanism of FOXD2-AS1/miR-185-5p/HMGA2 network in glioma via regulation of PI3K/Akt signaling pathway.

Methods: Microarray analysis was used for preliminary screening for candidate lncRNAs and mRNAs in glioma tissues. qRT-PCR and Western blot were used to determine the expression of FOXD2-AS1. The potential effects of FOXD2-AS1 on the viability, mobility and apoptosis of glioma cells were evaluated using MTT assay, Transwell assays and flow cytometry. The xenograft tumor model was performed to examine the influence of the lncRNA FOXD2-AS1/miR-185-5p/HMGA2 network on the biological functions of glioma cells. Luciferase assay and immunoprecipitation assay were examined to dissect molecular mechanisms.

Results: LncRNA FOXD2-AS1 was overexpressed in human glioma, and upregulated FOXD2-AS11 expression indicated higher WHO grade (p < 0.05). MiR-185-5p was downregulated, whereas HMGA2 was upregulated in glioma tissues in comparison with para-carcinoma tissues. FOXD2-AS1 could regulate the expression of HMGA2 via miR-185-5p. Knockdown of FOXD2-AS1 significantly inhibited proliferation and metastatic potential of glioma cells, whereas endogenous expression FOXD2-AS1 inhibited the glioma cell activity through targeting HMGA2.

Conclusions: lncRNA FOXD2-AS1 acted as a sponge of miR-185-5p and influenced the PI3K/Akt signaling pathway through regulating HMGA2. LncRNA FOXD2-AS1 modulated HMGA2 and PI3K/Akt downstream signaling through sponging miR-185-5p, thereby promoting tumorigenesis and progression of glioma.

The article "FoxD2-AS1 promotes glioma progression by regulating miR-185-5P/HMGA2 axis and PI3K/AKT signaling pathway" was retracted in 2023. Reasons: duplicated images; unreliable data; unreliable results or conclusions.

## Introduction

Glioma is one of the most common and invasive carcinomas in the central nervous system [1,2]. According to the WHO classification criterion, gliomas can be classified as grade I-IV based upon the pathological characteristics of malignant tumors. In spite of recent progress in cancer treatment, clinical prognosis and survival rate of glioma patients are still extremely low [3,4]. The malignant growth and high invasiveness of glioma cells severely constrain the therapeutic effect and cause a high recurrence rate [5]. Therefore, a better understanding of the key molecular mechanisms that mediate the development and progression of glioma will contribute to exploring novel and effective interventions.

Longnon-coding RNA (lncRNA) is constantly defined as an RNA that does not encode a protein, and the transcription length exceeds 200 nucleotides and lacks of the ability to encode a protein [6–8]. LncRNA HOXD-AS1 has been proven to be a carcinogen in human cancers [9–11]. At present, lncRNAs have been found to be abnormally regulated in various cancers [12]. Certain carcinogenic lncRNAs, such as H19, CAS C2 and HOTAIR have been identified to be poorly regulated [13]. It has been reported that lncRNA FOXD2-AS1 plays a pivotal role in tumor progression. For instance, Su et al. have found that FOXD2-AS1 promotes the progression and recurrence of bladder cancer through positive feedback loops of AKT and E2F1 [14]. Yang et al. have demonstrated that FOXD2-AS1 acts as a tumor promoter in colorectal cancer by regulating the EMT and Notch signaling pathways [15]. Chen et al. have proposed FOXD2-AS1 can promote the incidence of nasopharyngeal carcinoma by regulating the miR-363-5p/S100a1 signaling pathway [16]. However, the role and potential mechanism of FOXD2-AS1 in glioma remain elusive.

Consequently, the purpose of this study is to explore the exact role of lncRNA FOXD2-AS1 in pathogenesis of glioma and the potential mechanism underlying lncRNA FOXD2-AS1/miR-185-5P/HMGA2 signaling pathway in glioma.

## RESULTS

### Overexpression of lncRNA FOXD2-AS1 in glioma tissues and cells

The most significantly differentially-expressed lncRNA or mRNA were screened from the glioma and normal brain tissue samples according to the criteria of multiple change greater than 2 and *P*<0.05. In the glioma tissues, 285 lncRNAs were up-regulated and 483 lncRNAs were down-regulated. In the overexpression of lncRNA, the expression level of FOXD2-AS1 was up-regulated by 3.17 times on average. In addition, the expression levels of four lncRNAs were quantitatively detected by qRT-PCR and the results demonstrated that the expression levels of these lncRNAs in the glioma were significantly up-regulated than those in the adjacent tissues (Figure 1A, *P*<0.05). Among them, the expression level of FOXD2-AS1 was significantly up-regulated in low-/high-grade gliomas. HMGA2 plays a critical role in glioma progression [17]. Consistently, qRT-PCR revealed that HMGA2 was overexpressed in low-/high-grade glioma tissues (*P*<0.05, Figure 1B). Moreover, the expression levels of FOXD2-AS1 and HMGA2 were also significantly up-regulated in the U87 and U251 glioma cell lines compared with HEB cells (*P*<0.01, Figure 1C-D).

The article "FoxD2-AS1 promotes glioma progression by regulating miR-185-5P/HMGA2 axis and PI3K/AKT signaling pathway" was retracted in 2023. Reasons: duplicated images; unreliable data; unreliable results or conclusions.

**Figure 1:** **Expression levels of FOXD2-AS1 and HMGA2 were detected in glioma tissues and cells.** LncRNA expressions (**A**) and HMGA2 (**B**) in glioma tissues were examined by qRT-PCR. The expression of FOXD2-AS1 (**C**) and HMGA2 (**D**) in glioma cell lines was examined by qRT-PCR. *p < 0.05, **p < 0.01.

### LncRNA FOXD2-AS1 acts as a sponge of miR-185-5p

Bioinformatics analysis of potential miRNAs of FOXD2-AS1 was performed through online softwares, including StarBase v2.0 (starbase.sysu.edu.cn), miRcode (www.mircode.org) and miranda (www.microrna.org). The results revealed that FOXD2-AS1 contained complementary binding sequences of miR-185-5p seed regions (Figure 2A). RIP test results demonstrated that both FOXD2-AS1 and miR-185-5p could significantly enrich the miRNA ribonucleoprotein complex containing Ago2 (both *P*<0.01, Figure 2B, C), suggesting that FOXD2-AS1 and miR-185-5p belong to the same RISC complex. To further confirm the relationship between miR-185-5p and FOXD2-AS1, luciferase reporter vectors containing wt or mutant miR-185-5p binding sites in FOXD2-AS1 were constructed (Figure 2A) and co-transfected with miR-185-5p into HEK-293T cells. The results revealed that ectopic expression of miR-185-5 significantly down-regulated the luciferase activity of FOXD2-AS1-wt rather than FOXD2-AS1-mut (Figure 2D). Moreover, knockdown of FOXD2-AS1 significantly increased miR-185-5p expression in U251 and U87 cells (Figure 2E, F). However, transfection with miR-185-5p inhibitor had no significant effect on FOXD2-AS1 expression (Figure 2G, H). Together, these results suggest that FOXD2-AS1 interacts with miR-185-5p and negatively regulates miR-185-5p expression in glioma cells.

**Figure 2:** **LncRNA FOXD2-AS1 acts as a sponge of miR-185-5p.** (**A**) The wild type (wt) and mutant (mut) binding sites of miR-185-5p in FOXD2-AS1. (**B**, **C**) Relative expression levels of FOXD2-AS1 and miR-185-5p in U87 and U251 cells were detected by RIP assay. (**D**) U87 and U251 cells were co-transfected with FOXD2-AS1-wt (or FOXD2-AS1-mut) and miR-185-5p (or miR-control) and the luciferase activity was determined by the luciferase reporter assay. Control, non-transfected cells; NC, cells transfected with miR-control. **p < 0.01 vs. Control; ##p < 0.01 vs. NC. (**E**) Relative expression of FOXD2-AS1 after transfection with FOXD2-AS1 siRNA (si-FOXD2-AS1) in U251 and U87 cells was detected qRT-PCR. Control, non-transfected cells; si-NC, siRNA-control. **p < 0.01 vs. Control; ##p < 0.01 vs. si-NC. (**F**) Relative expression of miR-185-5p after knockdown of FOXD2-AS1 in U251 and U87 cells was detected qRT-PCR. Control, non-transfected cells; si-NC, siRNA-control. **p < 0.01 vs. Control; ##p < 0.01 vs. si-NC. (**G**) Relative expression of miR-185-5p after transfection with miR-185-5p inhibitor in U251 and U87 cells was detected qRT-PCR. Control, non-transfected cells; si-NC, siRNA-control. **p < 0.01 vs. Control; ##p < 0.01 vs. si-NC. (**H**) Relative expression of FOXD2-AS1 after inhibition of miR-185-5p in U251 and U87 cells was detected qRT-PCR. Control, non-transfected cells; NC, cells transfected with miR-control.

The article "FoxD2-AS1 promotes glioma progression by regulating miR-185-5P/HMGA2 axis and PI3K/AKT signaling pathway" was retracted in 2023. Reasons: duplicated images; unreliable data; unreliable results or conclusions.

### FOXD2-AS1 knockdown inhibits the proliferation and migration of glioma cells by regulating miR-185-5p

MTT assay showed that knockdown of FOXD2-AS1 significantly suppressed the growth of U251 and U87 cells. Inhibition of miR-185-5p blocked the effect induced by FOXD2-AS1 depletion. Moreover, suppressing miR-185-5p alone remarkably increased the cell viability of U251 and U87 cells (*P*<0.01, Figure 3A, B). Transwell assay showed that FOXD2-AS1 silencing dramatically reduced the cellular migration of U251 and U87 cells, whereas down-regulation of miR-185-5p effectively restored the migration capacity inhibited by FOXD2-AS1 knockdown. Additionally, downregulation of miR-185-5p alone markedly enhanced the migration ability of U251 and U87 cells (*P*<0.01, Figure 3C-F). We also detected the effect of FOXD2-AS1 on apoptosis. Flow cytometry analysis showed that FOXD2-AS1 knockdown remarkably enhanced the apoptosis in U251 and U87 cells, and treatment with miR-185-5p inhibitor restrained the apoptosis induced by FOXD2-AS1 silencing. Furthermore, treatment with miR-185-5p inhibitor alone significantly reduced the apoptotic rates of U251 and U87 cells (*P*<0.05, Figure 3G, H).

**Figure 3:** **FOXD2-AS1 regulates the proliferation, migration, and apoptosis of glioma cells by miR-185-5p.** (**A**, **B**) Effects of FOXD2-AS1 and miR-185-5p on the proliferation of U251 and U87 cells were detected by MTT. (**C**-**F**) Effects of FOXD2-AS1 and miR-185-5p on the migration of U251 and U87 cells were detected by Transwell migration assay. *p < 0.05, **p < 0.01 vs. Control; #p < 0.05, ^##^p < 0.01 vs. NC; ^&^P<0.05 vs si-FOXD2-AS1. (**G**, **H**) Effects of the FOXD2-AS1/miR-185-5p axis on the apoptotic rates of U251 and U87 cells were determined by flow cytometry. **p < 0.01 vs. Control; ^##^p < 0.01 vs. NC; ^&^p < 0.05 vs. si-FOXD2-AS1.

The article "FoxD2-AS1 promotes glioma progression by regulating miR-185-5P/HMGA2 axis and PI3K/AKT signaling pathway" was retracted in 2023. Reasons: duplicated images; unreliable data; unreliable results or conclusions.

### MiR-185-5p targets HMGA2

A binding site of miR-185-5p on HMGA2 3'UTR was observed by two bioinformatics programs, including miranda and TargetScan (Figure 4A). Luciferase assay demonstrated that the fluorescence intensity in the HMGA2-wt and miR-185-5p co-transfection groups was significantly decreased compared with that in the control group (both *P*<0.01), whereas no statistical significance was observed in the HMGA2-mut and miR-185-5p co-transfection groups (both *P*>0.05, Figure 4B), indicating a regulatory relationship exists between HMGA2 and miR-185-5p. Indeed, transfection with miR-185-5p mimic significantly reduced the protein and mRNA expression of HMGA2 (Figure 4C, D). In contrast, inhibition of miR-185-5p enhanced HMGA2 expression (Figure 4E-H). Moreover, treatment with miR-185-5p inhibitor remarkably abrogated the inhibitory effect of FOXD2-AS1 on HMGA2 protein expression (both *P*<0.01, Figure 4E, G). Similar results were also observed in the expression of HMGA2 mRNA as demonstrated by qRT-PCR (Figure 4F, H). Together, these results suggest that HMGA2 is a direct target of miR-185-5p.

**Figure 4:** **MiR-185-5p targets HMGA2.** (**A**) The binding site of miR-185-5p in the 3’UTR of HMGA2 was predicted via TargetScan. (**B**) Correlation between HMGA2 and miR-185-5p was validated in a luciferase reporter assay. (**C**, **D**) Protein and mRNA expression of HMGA2 after transfection with miR-185-5p mimic in U251 cells were analyzed by Western blot and qRT-PCR, respectively. (**E**-**H**) Effects of the FOXD2-AS1/miR-185-5p axis on HMGA2 protein (**E**, **F**) and mRNA (**G**, **H**) expression were analyzed by Western blot and qRT-PCR, respectively. **p < 0.01 vs. Control; ^##^p < 0.01 vs. NC; ^&&^p < 0.01 vs. si-FOXD2-AS1.

### FOXD2-AS1 regulates the proliferation and migration of glioma cells via miR-185-5p/HMGA2 axis

Next, we investigated whether the miR-185-5p/HMGA2 axis was critical for the function of FOXD2-AS1 in glioma cells. MTT assay showed that overexpression of miR-185-5p significantly inhibited the viability of U251 and U87 cells and this inhibitory effect was reversed by co-overexpression of HMGA2 (*P*<0.01, Figure. 5A-B). Transfection of HMGA2 alone markedly increased the growth of U251 and U87 cells (*P*<0.01, Figure. 5A-B). Transwell migration assays also demonstrated that co-transfection of miR-185-5p mimic and HMGA2 abolished the migration inhibition induced by miR-185-5p overxpression in U251 and U87 cells (*P*<0.01, Figure 5C, D). Overexpression of HMGA2 alone remarkably increased the growth of U251 and U87 cells (*P*<0.01, Figure 5C, D). Moreover, overexpression of HMGA2 restored the cell viability and migration ability of U251 cells inhibited by FOXD2-AS1 knockdown (*P*<0.01, Figure 5E, F). These results indicate that FOXD2-AS1 regulates the proliferation and migration of glioma cells through regulation of miR-185-5p/HMGA2 cascade.

The article "FoxD2-AS1 promotes glioma progression by regulating miR-185-5P/HMGA2 axis and PI3K/AKT signaling pathway" was retracted in 2023. Reasons: duplicated images; unreliable data; unreliable results or conclusions.

**Figure 5:** **FOXD2-AS1 regulates the proliferation and migration of glioma cells by miR-185-5p/HMGA2-mediated AKT signaling.** (**A**, **B**) The influence of miR-185-5p/HMGA2 axis on the proliferation of U251 and U87 cells was analyzed by MTT. (**C**,**D**) The effect of miR-185-5p/HMGA2 axis on the migration ability of U251 and U87 cells was analyzed by Transwell migration assay (200×). (**E**, **F**) Overexpression of HMGA2 abolished the inhibitory effects of FOXD2-AS1 on cell growth and migration in U251 cells as determined by MTT and migration assay. (**G**) Effects of the FOXD2-AS1/miR-185-5p/HMGA2 on the mRNA level of PI3K. (**H)** Effects of the FOXD2-AS1/miR-185-5p/HMGA2 on the levels of PI3K and phospho-Akt (p-AKT) in U251 and U87 cells were examined by Western blot. (**I**, **J**) Treatment of SC79 blocked the suppressive effects of FOXD2-AS1 on cell growth and migration in U251 cells. MTT assay and transwell assay were performed with transfected cells that treated with SC79 (5 µg/ml) for 48 h (I) and 24 h (**J**), respectively. **p < 0.01 vs. Control; ^##^p < 0.01 vs. NC; ^&&^p < 0.01 vs si-FOXD2-AS1.

### FOXD2-AS1 regulates PI3K/AKT signaling

qRT-PCR and Western blot results demonstrated that the mRNA and protein expression levels of PI3K and p-AKT were significantly down-regulated in the si-FOXD2-AS1 and miR-185-5p mimics groups, but dramatically up-regulated in the miR-185-5p inhibitor and p-HMGA2 groups (Figure 5G-H). Moreover, co-transfection with si-FOXD2-AS1 and miR-185-5p inhibitor reversed the down-regulation of PI3K expression and AKT phosphorylation induced by FOXD2-AS1 knockdown. On the other hand, co-expression of miR-185-5p and HMGA2 abrogated the inhibitory effects of miR-185-5p on levels of PI3K and p-AKT (Figure 5G-H). Furthermore, treatment with an activator of AKT, SC79 effectively blocked the suppressive effects of FOXD2-AS1 knockdown on cell viability and migration capability of U251 cells. Together, these results suggest that FOXD2-AS1 silencing inactivates PI3K/AKT signaling through the miR-185-5p/HMGA2 axis and thus suppresses the cell growth and migration of glioma cells.

### Knockdown of FOXD2-AS1 inhibits tumor growth in xenografts

To further investigate the effect of FOXD2-AS1 in vivo, a xenograft assay was performed. The results showed that the tumor volume and tumor weight in the si-FOXD2-AS1 group were significantly decreased compared with those in the control and NC groups (both *P*<0.01, Figure 6A-D). Moreover, qRT-PCR showed that the expression of miR-185-5p was significantly up-regulated in glioma tissues after FOXD2-AS1 silencing (*P*<0.01, Figure 6 E-F), which was consistent with the results found in U251 and U87 cells (Figure 2E, F).

The article "FoxD2-AS1 promotes glioma progression by regulating miR-185-5P/HMGA2 axis and PI3K/AKT signaling pathway" was retracted in 2023. Reasons: duplicated images; unreliable data; unreliable results or conclusions.

**Figure 6:** **The effect of FOXD2-AS1 on glioma growth *in vivo*.** (**A**-**D**) The effect of FOXD2-AS1 on glioma growth in mice injected with U251 (**A**, **C**) or U87 cells (**B**, **D**) transfected with sh-FOXD2-AS1 or sh-NC. (**E**, **F**) The effect of FOXD2-AS1 knockdown on miR-185-5p expression in glioma tissues of mice injected with U251 and U87 cells was analyzed by qRT-PCR. *p < 0.05, **p < 0.01 vs. Control; #p < 0.05, ##p < 0.01 vs. NC. Control, non-transfected cells; sh-NC, cells transfected with shRNA-control.

## DISCUSSION

Previous results have demonstrated that the pathogenesis of glioma requires the changes in multiple genetic pathways, and each primary and secondary glioma possesses a unique combination of these genetic changes [18]. Primary glioma is constantly characterized with loss of heterozygosity at 10q (LOH, 70%), EGFR amplification (36%), deletion ofp16INK4a (31%) and mutation of PTEN (25%) [17]. In our study, we focused on lncRNA FOXD2-AS1, which has been found to be aberrantly expressed in various cancers. In this experiment, lncRNA FOXD2-AS1 was highly expressed in human glioma tissues and cell lines. Next, we investigated the downstream molecular mechanism of FOXD2-AS1 in glioma. In this study, we found a regulatory relationship between lncRNA FOXD2-AS1 and miR-185-5p, and between miR-185-5p and HMGA2. Compared with adjacent normal tissues, the expression of miR-185-5p was down-regulated, whereas the expression of HMGA2 was up-regulated in glioma tissues. In addition, HMGA2 overexpression had the potential to promote the proliferation and migration of glioma cells, whereas miR-185-5p mimics inhibited the biological function of glioma cells by targeting HMGA2. Finally, lncRNA FOXD2-AS1 was proven to act as the sponge of miR-185-5p and affects the PI3K/AKT signal transduction pathway via regulating HMGA2.

Recent evidence has suggested that FOXD2-AS1 silencing can inhibit malignant biological behavior of cancer cells. For instance, Zhu et al. revealed that FOXD2-AS1 knockdown can weaken the malignant behavior of colorectal cells by inhibiting cell migration and invasiveness [19]. Bao et al. have also confirmed that the high expression of FOXD2-AS1 is correlated with the poor prognosis of patients diagnosed with esophageal squamous cell carcinoma [20]. Besides, lncRNA can serve as a competitive endogenous RNA sponge for miRNA to regulate the degradation of miRNA target, thereby affecting the post-transcriptional regulation in bladder cancer [21]. In the present investigation, we first screened out the significantly differentially-expressed lncRNAs based on microarray assay and lncRNA FOXD2-AS1 was highly expressed in glioma. Subsequently, bioinformatics analysis, luciferase reporter gene assay and RIP test were conducted to confirm the regulatory relationship between FOXD2-AS1 and miR-185-5p. The findings of this study further validate that the transcriptional activation of FOXD2-AS1 contributes to tumorigenesis, whereas FOXD2-AS1 knockdown impairs the carcinogenic function of miR-185-5p in glioma cells.

The article "FoxD2-AS1 promotes glioma progression by regulating miR-185-5P/HMGA2 axis and PI3K/AKT signaling pathway" was retracted in 2023. Reasons: duplicated images; unreliable data; unreliable results or conclusions.

It has been reported that HMGA2 plays a role in carcinogenesis and up-regulation of HMGA2 triggers the migration of cancer cell population via activation of PI3K/AKT downstream signal transduction [22]. In addition, previous studies have demonstrated that the expression of PI3K/AKT is up-regulated in glioma. In most circumstances, the loss of PI3K inhibitor PTEN (phosphatase and tens in homologue) or the functional acquisition mutation of PI3KCA5 is a potential cause. In the current study, we explicitly elaborated the regulatory mechanism of FOXD2-AS1/miR-185-5p pathway upon the HMGA2 and PI3K/AKT signaling pathways, and eventually demonstrated that FOXD2-AS1 promoted HMGA2 by suppressing miR-185-5p, thereby regulating the proteins of PI3K and p-AKT. A diagram summarizing the main findings of this study was shown in Figure 7. In this study, the expression levels of PI3K and p-AKT were significantly down-regulated in the si-FOXD2-AS1 and miR-185-5p mimics groups, whereas considerably up-regulated in the miR-185-5p inhibitor and p-HMGA2 groups, indicating that FOXD2-AS1 regulates the PI3K/AKT signal pathway through the miR-185-5p/HMGA2 axis.

**Figure 7:** A diagram summarizing the main findings of this study and illustrating the complex regulatory relationship of the lncRNA/microRNA/mRNA network and epigenetic regulation pathways.

## Conclusion

Taken together, lncRNA FOXD2-AS1 and HMGA2 are overexpressed in glioma tissues and cell lines. A regulatory relationship exists between miR-185-5p and lncRNA FOXD2-AS1 or HMGA2. Moreover, lncRNA FOXD2-AS1 acts as a sponge of miR-185-5p to regulate HMGA2 expression and PI3K/AKT signaling pathway and subsequently promote the occurrence and progression of glioma. The findings in this study not only contribute to in-depth exploration of the exact mechanism of lncRNA FOXD2-AS1, but also provide a promising therapeutic target for the treatment of glioma.

The article "FoxD2-AS1 promotes glioma progression by regulating miR-185-5P/HMGA2 axis and PI3K/AKT signaling pathway" was retracted in 2023. Reasons: duplicated images; unreliable data; unreliable results or conclusions.

## MATERIALS AND METHODS

### Patients and samples

Human glioma samples were collected from 48 glioma patients (31 males and 17 females) who underwent neurosurgery in the Department of Neurosurgery of the Third Affiliated Hospital of Kunming Medical University from January 2013 to October 2015. Normal brain tissues were obtained from 24 patients with brain injury who were randomly selected from 2014 to 2016 and underwent brain tissue resection. All samples were restored in liquid nitrogen, and all participants did not receive radiotherapy before the experiment. Clinical parameters of glioma patients were shown in Supplementary Table S1. Written informed consents were obtained from all participants. The study procedures were approved by the Ethics Committee of the Third Affiliated Hospital of Kunming Medical University.

### Cell culture and reagent

Human glioma cells (U87, A172, U251 and T98G) and normal cells (HEB) were purchased from BeNa Culture Collection (BNCC, Beijing, China). All cells were cultured in Dulbeco’s modified Eagle medium (DMEM, Gibco, Thermo Fisher Scientific) supplemented with 10% fetal bovine serum (Sigma-Aldrich, St.Louis, MO, USA) at 37°C and 5% CO_2_. SC79 was purchased from Sigma-Aldrich (Louis, MO, USA) and dissolved in dimethyl sulfoxide (DMSO).

### Microarray analysis

The Gene Expression Omnibus (GEO) database was utilized to screen the differentially expressed lncRNAs and mRNAs from tumor and normal tissues. The Blimma tool kit in the R script was adopted to identify differentially expressed genes under experimental conditions. The microarray data were subjected to logarithmic transformation, Benjamini-Hochberg adjust method [23] for Bayesian test. The differentially expressed genes were screened using multiple changes (*P*<0.05, |log (multiple changes) |>2).

### qRT-PCR

Total RNA was extracted from frozen tissues or cultured cell lines using TRIZOL reagent (Life Technologies, Carlsbad, CA). The total RNA was reverse-transcribed into cDNA using the ProtoScript® First Strand cDNA Synthesis kit (New England Biolabs, Ipswich, MA, USA). qRT-PCR was performed using fluorescence quantitative PCR. The primer sequences were illustrated as follows: MiR-185-5p, F: 5′-TGAGGAGCCGATCACGTC-3′, R: 5′-GTGCCGGTGCAGAGGT-3′; FOXD2-AS1, F: 5′-CTCACATCCGGCGGCT-3′, R: 5′-GGCTGTTCATGATATGTGCCA-3′; HMGA2, F: 5′-ACACTGTCCTGACAACTGCC-3′, 5′-AGGGGTGTGGGTGGTATTCT-3′; PI3K, F: 5′-CTCTCCTGTGCTGGCTACTGT-3′, R: 5′-GCTCTCGGTTGATTCCAAACT-3′; GAPDH, F: 5′-CCTGACCTGCGTGTGGACT-3′, 5′-GCTGTGGATGGGGAGGTGTC-3′. The relative expression was standardized by GAPDH and the multiple changes were measured by 2-ΔΔCt method.

The article "FoxD2-AS1 promotes glioma progression by regulating miR-185-5P/HMGA2 axis and PI3K/AKT signaling pathway" was retracted in 2023. Reasons: duplicated images; unreliable data; unreliable results or conclusions.

### Plasmid generation

The FOXD2-AS1 sequence was synthesized and subcloned into the pCDNA3.0 (Invitrogen, Shanghai, China) vector. The experimental design was divided into 8 groups: the control (empty vector), negative control (NC, Scrambled control), siRNA-FOXD2-AS1 (si-FOXD2-AS1), pcDNA3.0-HMGA2 (p-HMGA2), miR-185-5p inhibitor, miR-185-5p mimics, miR-185-5p inhibitor + si-FOXD2-AS1 and miR-185-5p mimics + p-HMGA2. Glioma cells were inoculated into a 6-well plate. Cell transfection was carried out according to the Lipofectamine 2000 instructions.

### Dual-luciferase reporter assay

Dual-luciferase reporter assay was performed to investigate the regulatory relationship between lncRNA FOXD2-AS1 and miR-185-5p, as well as the relationship between HMGA2 and miR-185-5p. The FOXD2-AS1 (or HMGA2 3'UTR) fragments containing the predicted wild-type (wt) or mutant (mut) miR-185-5P binding site (RiboBio Co., Ltd. Guangzhou, China) were cloned into pmirGLO vector (Promega, Madison, Wisconsin, USA). To determine the luciferase activity, HEK-293T cells were seeded in a 96-well plate. The 50 nM pmirGLO-FOXD2-AS1-wt (or pmirGLO-HMGA2-wt) or pmirGLO-FOXD2-AS1-mut (or pmirGLO- HMGA2-mut) were co-transfected with 50 nM miR-185-5p or miR-control (NC) by using Lipofectamine 2000 (Invitrogen). The luciferase activity was measured using the dual-luciferase reporter gene subsystem according to the manufacturer’s instructions (Promega, Madison, Wisconsin, USA).

### RNA immunoprecipitation

The RNA immunoprecipitation (RIP) test was conducted using the Magna RIP RNA-binding protein immunoprecipitation kit (Millibo, Billyka, MA, USA) according to the manufacturers’ protocols. The U87 and U251 cells were lysed using a complete RIP lysis buffer, and 100 μl of the whole cell extract was incubated with RIPA buffer containing human anti-Argonaute 2 (AgO2) antibody (Millipore)-conjugated magnetic beads (#AK6979) at 4°C for 6-8 h. Normal mouse IgG (Millipore) was used as negative control.

### MTT assay

Cells were seeded into a 96-well plate and incubated at a density of 5×10^3^ at 37°C. After cell incubation for 0, 24, 48 and 72 h, MTT was supplemented into each well. The mixture was incubated at 37°C and 5% CO_2_ for 4 h, supplemented with 150 mL DMSO and dissolved at room temperature for 20 min. The absorbance value of each well was measured at a wavelength of 490 nm by an ultraviolet spectrophotometer.

### Apoptosis analysis

The cells were seeded in a 6-well plate for 24 h. The cell apoptosis was detected by using Annexin V-FITC/PI apoptosis detection kit according to the manufacturers’ instructions (BD Biosciences). The mixture was then shaken thoroughly in a dark room at room temperature for 15 min and supplemented with 2.5 μL PI. Cytomics FC 500 flow cytometer was adopted to analyze cell apoptosis.

The article "FoxD2-AS1 promotes glioma progression by regulating miR-185-5P/HMGA2 axis and PI3K/AKT signaling pathway" was retracted in 2023. Reasons: duplicated images; unreliable data; unreliable results or conclusions.

### Transwell assay

Transwell filter (BD Biosciences) was employed to perform Transwell migration as previously described [24].

### Western blot

Protein extraction and Western blot were carried out as described below. The rabbit polyclonal antibody against HMGA2 (cat#5269, 1: 500), rabbit polyclonal antibody against PI3K (cat#9272, 1: 500), rabbit polyclonal antibody against P-AKT (cat#4058, 1: 500), PI3K (cat#4292, 1: 500) and mouse monoclonal antibody against GAPDH (Cat#9662, 1: 500) were purchased from Cell Signaling Technology. After overnight incubation at 4°C, the membrane was washed with TBST for three times and incubated with horseradish peroxidase-conjugated goat anti-mouse IgG secondary antibody or horseradish peroxidase-conjugated goat anti-rabbit IgG (1: 2000). Western blot was determined using ImageJ2X software (National Institutes of Health, Bethesda, Maryland, USA).

### Tumor xenograft transplantation

Four-week-old speciﬁc pathogen-free (SPF) BALB/c nude mice were selected and divided into 6 groups. After 1-week adaptation, approximately 5×10^6^ U251 or U87 cells transfected with NC, shNC, sh-FOXD2-AS1, NC, mimics-NC or miR-185-5p mimics were subcutaneously inoculated into the right side of the mice in each group (n=8). The volume was measured every week and calculated using the following formula: Volume (cm^3^) = (length × width^2^)/2. After 4 weeks, the mice were sacrificed. The tumor tissues were extracted and prepared for subsequent experiment. This study was approved by the Ethics Committee of Animal Experiment Center of the Third Affiliated Hospital of Kunming Medical University.

### Statistical analysis

All data were presented as mean ± SD. All statistical analyses were performed by SPSS statistical software 17.0 (SPSS Inc., Chicago, IL, USA) and GraphPad Prism software (version 5.0). Group comparison was conducted by using Student’s *t*-test or one-way ANOVA. The relationship between FOXD2-AS1 level and clinicopathological features was determined by χ2 test. *P*-values of statistical significance are represented as *P<0.05, **P<0.01 and ***P<0.001.

## Supplementary Material

Supplementary Table
